The article "Quantitative Evaluation and Optimal Decision-Making Study on the Cultivation under the Environment of Humanistic Literacy Based on Advanced Data Analysis Technologies" was retracted in 2023. Reasons: signs of a paper mill; suspected computer-generated content; unreliable results or conclusions; lack of ethics approval or compliance.

# Quantitative Evaluation and Optimal Decision-Making Study on the Cultivation under the Environment of Humanistic Literacy Based on Advanced Data Analysis Technologies

**DOI:** 10.1155/2022/8918871

**Published:** 2022-09-29

**Authors:** Shengru Meng

**Affiliations:** ^1^School of Education, Tianjin University, Jinnan, Tianjin 300350, China; ^2^Hainan University, Haikou, Hainan 570228, China

## Abstract

As an important part of China's higher education, higher vocational education occupies an extraordinarily important position in China's higher education system. In order to clarify the literacy of higher vocational students, carry forward their excellent quality, and correct their bad habits, a quantitative evaluation and optimization decision-making research on the cultivation of humanistic literacy of higher vocational students based on data mining technology is proposed. By using data mining technology, the important data of students can be obtained quickly; by using advantages of information integration, the cultivation of humanistic quality of higher vocational students is evaluated from a correct perspective; by strengthening the education of campus culture construction, students' moral quality can be enhanced, students' enthusiasm for learning can be mobilized, the advantages of new media's public opinion orientation can be given full play, and a humanistic and healthy growth environment for vocational students can be created. Through experiments, it is proved that data mining can better evaluate the humanistic quality of students. During the learning process, the humanistic quality evaluation of female college students reaches 95%, and the overall quality of male and female gradually rises to 80%.

## 1. Introduction

After entering the 21st century, Chinese higher education circles generally [1] realized that quality of general education, moral quality, and quality of professional skills are the three most important qualities that contemporary college students should possess, and at the same time, they began to use large-caliber professional education to locate and plan higher education with general education as the base. Education is to help people educated develop their abilities [2], perfect their personality, and fulfill their responsibilities in human culture. General education is the education of developing perfect people, multifaceted people, and people with the sound personality. Education is a noble moral education. Humanistic training is the core of general education [3], which crosses throughout the whole process of integrating general education into overseas education in domestic and foreign universities [4]. Therefore, rich connotation is one of the characteristics of general education, which can be understood from three levels of educational philosophy, educational content, and talent training model [5]. The concept of general education in all countries is the same, with the cultivation of sound talents as the main content, the cultivation of “returning to people themselves” as the purpose, and the cultivation of “all-round quality” talents as the benchmark purpose [6]. The focus of the research is the construction of humanistic spirit and comprehensive quality. The goal of general education is to make college students in a country have a common knowledge system and cultural background [7].

What is humanistic literacy? Literally, it refers to the research ability, knowledge level of the humanities, and the people-oriented spirit embodied in the humanities, that is, the inherent quality of people. In other words, humanistic literacy has two meanings: one is the knowledge level; that is, there must be a certain reserve of humanistic knowledge [8]; the other is the spiritual level; that is, there must be a certain humanistic quality, which can be a sense of social moral responsibility, independent thinking ability, or a quality of sympathy and compassion for the weak and tolerating and helping others. Among the two, the former is the foundation, and the latter is the core, and both are indispensable. After all, knowledge and experience are the source and motivation of spirit [9], and spiritual quality is the external manifestation of knowledge cultivation. Only under the interaction of the two can students' huge energy be burst out, so that they can better adapt to future work and life, can calmly analyze problems in a comprehensive and in-depth manner, and can be tolerant and friendly for others, which truly reflects the achievements and functions of higher education. However, the current situation of humanistic quality of vocational students is not optimistic, especially in the spiritual level. Therefore, on the basis of digging deeply into the causes of this phenomenon, the essence must be seen through the phenomenon [10], and a reasonable solution must be sought.

In view of the drawbacks of the traditional physical and chemical experimental evaluation system, literature [11] carried out new design and practice in terms of evaluation methods, evaluation contents, and evaluation standards. Establishing a new evaluation system is an effective way to improve teaching quality and cultivate and promote students' comprehensive design ability and innovation ability. Based on career belt theory, policy documents, and core career competencies, literature [12], starting from the three dimensions of knowledge, professional ability, and basic professional quality, clarified the connotation and weight of evaluation indicators and provided some suggestions for evaluating students. Literature [13] evaluated the curriculum reform of basic education through the cultivation of students' comprehensive quality, further studied the evaluation standards, improved the evaluation plan, created an evaluation environment, strengthened the cultivation of evaluation subjects, and cultivated students' comprehensive quality on the basis of professional practice. In accordance with the concept of quality education, literature [14] deepened the connotation of the comprehensive quality of college students, focused on the optimization and upgrading of the comprehensive quality structure of college students, and promoted the implementation of quality education reform [11–14]. To sum up, the aforementioned research focuses on other aspects of students' literacy, and the evaluation results are relatively good, but it does not focus on the study of humanistic literacy. Therefore, this paper evaluates the humanistic literacy of higher vocational students and formulates an optimization plan.

The cultivation of humanistic literacy can help students form a correct world outlook, outlook on life and values. The cultivation of vocational ability should be the primary task of higher vocational education [15]. Its essence is to realize the prosperity of the country, the rejuvenation of the nation, and the happiness of the people and to connect the country, the nation, and the people. How to realize the Chinese dream is to stick to the Chinese road, carry forward the Chinese spirit, and rely on Chinese strength [16]. The Communist Party of China has put forward the goal of realizing the great rejuvenation of the Chinese nation. As the builders and successors of socialism with Chinese characteristics and the backbone of realizing the Chinese dream, contemporary college students are required to have a good attitude [17]. With increasingly improved material conditions [18] and more prominent spiritual needs, the cultivation of humanistic quality of college students in higher vocational colleges reflects the care for people [19]. To stimulate students' awareness of life value and better meet the needs of students' all-round development is an inevitable requirement for Chinese economic and social development in new stage. At the same time, it is also obvious that as the educational concept of quick success and pragmatism is constantly developing and becoming stronger, schools, families, and society will inevitably suffer from the drawbacks and adverse consequences of utilitarian education [20]. Quick success and pragmatism education ignores students' all-round development and the cultivation of humanistic qualities, which not only damages students' own health and happiness and inhibits students' innovative potential [21] but also leads to the lack of students' social responsibility, honesty quality, hard-working spirit, cooperation awareness with others, etc. [22]. Some students in higher vocational colleges pay too much attention to the immediate opportunities and the development of material and spiritual relationships [23], ignoring the great ambitions and goals. They pursue hedonism without taking into account their own characteristics and realities, personal development, and career prospects. School education is the foundation and hope for improving the quality of a nation. Putting fostering characters and civil virtues in the first place, campus education should pay attention to students' humanistic quality, strengthen the cultivation process of humanistic literacy, and promote students' all-round development, so that the younger generation can make new contributions to the establishment of national image and world civilization [24].

Vocational colleges are an important part of Chinese higher education system. The demand for skilled talents in economic development is the top priority of higher vocational colleges. With the development of the times and the reform of the society, the employment concept in the past is no longer suitable for the development of today's society. In particular, the socialist ideology with Chinese characteristics in the new era requires highly skilled and high-quality talents. Therefore, higher vocational colleges must keep pace with the times. As a vocational college, in the face of the current situation of popularization of vocational education, how to make students have innovative spirit and high-level humanistic quality and how to improve students' communication skills, information processing skills, critical thinking skills, and logical analysis skills are the starting point for cultivating students. Improving humanistic quality plays an important role in vocational students' overall development and world outlook, view of life, and value education, which is able to broaden students' horizons, promote knowledge and cultural exchanges with companies around the world, and lay a solid foundation for college students to start their own businesses. This paper is based on the data mining technology to establish the classification data model of students' humanistic literacy evaluation. First of all, several nodes correspond to teaching quality attributes one by one. Then, the node branches are used to represent the value judgment of each attribute, and finally, the classification results are used to evaluate students' humanistic quality and complete the quality optimization.

## 2. Theoretical Overview of Data Mining

Data mining technique originates in the fields of statistics [25, 26], databases, and machine learning. Its main task is to mine useful knowledge or discover potentially [27] valuable relationships from large amounts of data. Knowledge in data mining refers to the information hidden in data. By mining and exploring this latent knowledge from large amounts of unprocessed data, it is ultimately made available to managers or analysts for decision support. Data mining technique [28] is based on many disciplines, including ergonomics [29], pattern recognition, and visual analysis techniques.

There are two main categories of tasks in data mining. The first is the prediction of unknown things [30]. The other is to automatically partition large amounts of unlabeled data and automatically cluster similar content together.

Classification is mainly to classify new things. The classifier must first have a labeled data set and then uses a data set as a training set to build various classification models on this training set so as to classify the unknown things. Currently, there are many successful classifiers such as decision trees, naive models, artificial neural networks, and support vector machines. All of these algorithms can perform classification, and some can build good structural models that explain the entire data set well.

The task of clustering is to automatically aggregate large amounts of data. Cluster analysis techniques have been used in many research fields to automatically group similar things together. For example, in psychology, clustering techniques are used to study the causes of depression; in biology, clustering techniques are used to automatically classify organisms; and in information detection, clustering techniques are used to group similar web pages together.

After years of exploration and research, people have summarized the basic process of data mining technology. It involves cleaning, extracting, and transforming the required data from the uncleaned raw data, generating a data set, building a classification or clustering model based on the data set, and finally extracting and analyzing the information. The specific flow is shown in Figure 1.

In order to make the data more real and have a certain value, it is necessary to find methods and ways to make the application of data mining technology more widely promoted. Data is a huge information resource base, and some characteristics or laws can be grasped by studying and mining the resource information in the data. Here are some information analysis methods.

### 2.1. Correlation Analysis Method

Things are always related, and so the data are. Since the amount of information in the data is very large and it takes a long time to find its correlation, it is difficult to find the rules between the data. To improve the efficiency and accuracy of finding data correlations, correlation analysis method is adopted, which can use data parsing tasks to help people improve efficiency and quality. Due to its strong purpose, this method can be used for information management with high data accuracy.

### 2.2. Cluster Analysis Method

The so-called clustering is to group and classify different data and convert scattered data into organized information. However, clustering is not only a common classification method but can find meaningful data information in a data set without knowing the objects. Therefore, the disadvantage of this method is that it cannot accurately classify data information, which is the reason why this method is only used in psychology, data recognition, and other fields.

### 2.3. Characteristic Analysis Method

With the advent of the era of data explosion, classified data also needs to be based on its own characteristics. This method is to obtain effective information according to the characteristics of the data. For example, computer methods are used to classify virtual data of data, find out the characteristics of data, and use the analysis results to perform classification.

### 2.4. Artificial Neural Network

The method belongs to the above-mentioned feature analysis method; that is, a large amount of data is first processed; then, a network model is established for these data, and finally, a neural network is used to analyze the data.

### 2.5. Quantitative Evaluation Method

The so-called quantitative evaluation refers to transforming the evaluation content into a specific “quantity” form and investigating, collecting, and analyzing relevant data to achieve the purpose of effective evaluation and comprehensive evaluation. At present, the comprehensive evaluation method formed by higher vocational colleges under the guidance of quantitative evaluation is the credit system, which is used to quantitatively evaluate the humanistic quality of vocational students.

### 2.6. Data Mining Method

Data mining mainly consists of three steps: forming quantitative evaluations, obtaining a library of conditional patterns, and optimizing decisions. The task of the insertion stage is to form quantitative evaluation, which is used to obtain a library of conditional patterns in the next stage and conduct optimization decisions in the last stage.

## 3. Optimization of the Cultivation Path of Humanistic Literacy of College Students in Higher Vocational Colleges

### 3.1. Strengthen the Construction of Campus Culture to Realize Cultural Education

Campus cultural activities can be said to be the second classroom for college students, which is the activity base for college students in higher vocational colleges to accept humanistic literacy. Strengthening the education of campus culture construction is conducive to giving play to the dominant position of higher vocational students, cultivating humanistic spirit, and improving the humanistic quality of higher vocational students. To this end, schools should set up various social groups and hold various forms of humanistic quality practice activities to enrich students' humanistic knowledge and cultivate students' humanistic spirit in practice. Campus social groups can hold humanities, culture, and social science lectures, invite well-known scholars and experts to give humanities academic reports, and use special festivals to hold cultural art festivals and theme education activities, so as to carry forward traditional culture and improve the moral quality of college students' humanistic quality. Campus media can create a public opinion atmosphere of university spirit in various ways. The content disseminated by the campus media can be conductive to propagandizing fighting thoughts or promoting the learning of young people. These are the continuation of the classroom and the sublimation of knowledge and are effective means to cultivate college students' humanistic knowledge and humanistic spirit. On the other hand, the campus library primarily has rich and complete book resources, various reading forms, and huge reserves of electronic network information resources. Therefore, the university library can also play its role as a higher education base for higher vocational colleges, collecting some books on the humanities and social sciences such as literature, history, and philosophy. These books are the crystallization of traditional Chinese culture, with high artistic charm and cultural connotation, which are the material guarantee for college students to improve their humanistic quality.

### 3.2. Establish a “People-Oriented” Educational Concept and Clarify Educational Goals

The 21st century is an era of rapid development of science and technology. The strength of international competitiveness depends on the level of science and technology. Therefore, China proposes that science and technology education plays a fundamental role in the formation of comprehensive national strength. The strength of comprehensive national strength depends on the quality of laborers and talents, and the cultivation of talents depends on education. Since the reform and opening up, education in China has made remarkable achievements. Continuing to deepen education reform and comprehensively promoting humanistic quality education to lay a solid talent and knowledge foundation for the implementation of the strategy of rejuvenating the country through science and education and the strategy of strengthening the country through talents is a constant policy. To carry out humanistic cultivation is to establish the educational concept of “people-oriented,” which is the core of the scientific development concept, the unity of values and methodology, and the connotation of educational philosophy and political philosophy. For this, the fundamental task of colleges and universities is to develop their own academic beauty, moral beauty, intellectual beauty, healthy beauty, and physical beauty in an all-round way, so as to realize the harmony and unity of training goals and the optimal development of personality. Secondly, it is necessary to respect the dominant position of students in the process of education and teaching, respect the independent personality of students, and give students the initiative in learning. Thirdly, the enthusiasm of teachers in educational practice, the initiative of teaching practice, and the creativity of teachers' educational practice should be given full play, so as to guide students in higher vocational colleges to carry out self-education and fully mobilize students' enthusiasm for learning.

### 3.3. Optimize the Social and Cultural Atmosphere and Give Full Play to the Advantages of New Media Public Opinion Orientation

To optimize the social and humanistic quality atmosphere, the cultural and educational functions of the society should be first given full play. For instances, guided by the advanced socialist culture, it is feasible to guide students to form cultural awareness and sense of responsibility, enrich the campus cultural life of college students with elegant culture, improve the aesthetic and artistic ability of college students, promote social mainstream values, guide the society to form a positive social atmosphere and positive energy, and effectively utilize the cultural leading role of museums, memorial halls, cemeteries, exhibition halls, etc., in the patriotic education base. Meanwhile, to cultivate the patriotism, good moral character, and innovative spirit of college students in higher vocational colleges, new media should promote mainstream values, guide college students with correct public opinion, and adhere to the unity of knowledge and interests, as well as the unity of economic and social benefits. Only in this way can the discrimination ability of college students in higher vocational colleges be improved to establish correct human values and world outlook and can their own humanistic quality be perfected. Today's world is an era of rapid development of the Internet. College students are the group that contacts and uses the Internet the most and also the group that is most affected by the Internet. Therefore, network management departments at all levels should strengthen network governance, establish green websites, strengthen network ethics education, guide mainstream thinking, use strict and effective technical means to resist network spam and bad information, purify the network environment, and spread positive energy, so as to serve the higher vocational colleges and create favorable conditions for college students to achieve humanistic and healthy growth.

## 4. Experiment and Analysis of Experimental Results

Based on the teaching-related data in the educational administration system, this paper establishes a basic data model consisting of attributes such as student ID, student name, gender, grade, and class. After data transformation and loading, data mining is used to calculate the attributes which are the most relevant to performance analysis and evaluation features, and then, an iterative recursive method is used to classify the remaining attributes and build a model.

First of all, a student data table is established, which contains the student's name, age, gender, grade, major, and some basic information. By analyzing the following information, the relationship between the quality indicators can be evaluated, which is shown in Table 1.

The test results are divided into three grades: A grade is the range of 80 points and above, B grade is the range of 70 to 80 points, and C grade is the range of 70 points or less, which are used as indicators for evaluating students' humanistic literacy. Then, a classification model is established to describe students' humanistic literacy, and the evaluation results of teaching quality are formed according to the scores. At the same time, using the classification model formed by the decision tree, the IF-THEN classification rules are formed.

Then, according to the students' humanistic quality requirements, a questionnaire is established. The specific contents include the following points:

1. Actively prepare class content
2. Strictly implement work and rest time, and there is no lateness or early departure
3. Have a correct and serious learning attitude
4. Respect teachers and leaders, and there is a harmonious relationship between teachers and students
5. Learn to enrich humanistic knowledge and cultivate humanistic spirit in practice
6. Improve the aesthetic and artistic ability of college students
7. Hold cultural and artistic festivals and themed educational activities to promote traditional culture
8. The learning method is flexible, full of passion, and can infect the teaching process
9. Have strong learning and innovation ability
10. Be able to really learn the corresponding knowledge and skills

In view of the above assessment content, a questionnaire in the form of single-choice and multiple-choice is prepared. 200 students in each grade are surveyed, and the responses are authentic, valid, and persuasive. In order to facilitate the next data processing, combined with the content of the questionnaire and the relevant teaching evaluation standards, the four levels of A, B, C, and D are divided, in which A is the best, and D is the average. Then, the 200 pieces of questionnaires are divided into different grades to form an evaluation information table.

According to the data analysis requirements of this teaching quality assessment, this paper uses Tomcat 6.0 to build a network server, designs and develops a platform through Eclipse Jee-Mars, and embeds the associated data into the assessment platform through data mining technology, so as to analyze and find out the association rule data items that are valuable for the evaluation of students' humanistic quality. By filtering and sorting, several valuable rules are listed:

Rule 1: correlation between age and evaluation scores: all scores above the age of 18 are “excellent”

Rule 2: correlation between gender and evaluation scores: all the scores of females are “good”

Rule 3: correlation between professional categories and evaluation scores: through the analysis of relevant data, there is no necessary relationship between students' professional categories and the evaluation of humanistic quality

According to the above rules, from the 200 questionnaires, it is concluded that with respect to gender, the evaluation of female students in higher vocational colleges is generally high, and the data reaches 95%, which indicates that women's literacy is better; with respect to age, 80% of students are more mature in their studies, paying more attention to speech and behavior; while with respect to professionalism and literacy, 90% have no relationship.

Finally, 200 students aged 16-20 years old are selected from higher vocational students as research objects, including 100 men and women, and the remaining data should not be regarded as important conditions. On the first day, 200 students are evaluated for humanistic quality, and after 30 days of course training and educational activities, the optimization effect of students is judged.

As can be seen from Figure 2, without quality optimization, the humanistic quality of male and female students is generally lower than 90 points, and the low segment of male students is hovering between 60 and 70 points, and the score of female students is hovering between 80 and 90 points. When the number of male students before optimization is 100, the lowest score is 60 points; when the number of male students is 20, the highest score is 70; when the number of female students before optimization is 40, the highest score is 87 points; when the number of female students before optimization is 60, the minimum score is 82 points. After 30 days of course training and quality education activities, it can be seen that the humanistic quality of male and female students has been greatly improved, and the score of male students has increased to between 75 and 80 points. When the number of male students is 10, the score reaches 80 points, with the best optimization effect; when the number of male students is 100, the optimization effect takes second place. In contrast, the score of female students improves significantly in the 90-100 score range. When there are 60 female students selected, the highest score is 100 points, with the best optimization effect.

Figure 3 shows that in the 16-20 age group, after 30 days of course training and educational activities, the score of 16-year-old students before the cultivation of humanistic literacy is lower than 55 points, and 17-year-old students have a lower score of 60 points. Meanwhile, the score of 18-year-old students before humanistic literacy training is around 65 points, the score of 19-year-old students before humanistic literacy training is 70 points, and the score of 20-year-old students before humanistic literacy training is the highest of 75 points. After another 30 days of courses, 16-year-old students have reached 80 points from the previous 55 points, 17-year-old students have reached 85 points from 60 points, 18-year-old students have achieved 90 points from 65 points, 19-year-old students have reached 95 points from 70 points, and 20-year-old students have the highest score improvement, which can reach 100 points. It can be concluded according to the figure that a large part of the humanistic quality evaluation of students in each age group has improved, and in particular, the optimization effect is obvious for older students.

The era of big data is mostly characterized by highly developed information. Mining and integrating valuable huge information groups is actually exploring and applying data mining technology in the era of big data. Using the method of data mining can not only satisfy the changing role of data in daily information management but also deal with the trouble of mutual interference of information. In order to provide development resources for the cultivation of humanistic literacy of higher vocational students, it is necessary to dig and explore the hidden data and information, integrate these data and information, and make plans for the next use, so as to make the information resources effective. Moreover, reasonable and effective use of data mining technology also enables resource information achieve optimal use effect.

## 5. Conclusions

In the era of big data, the application of data mining not only facilitates to people's life but also improves people's quality of life. Data mining technology is well integrated into various fields to provide convenient and high-quality services for various fields, so as to meet the needs of this era. From the perspective of cultivating the humanistic quality of higher vocational students, based on the decision tree technology of data mining, this paper establishes a data model for the classification of students' humanistic quality evaluation and constructs a humanistic quality training optimization strategy that is more in line with the needs of society, enterprises, and students. At the same time, the construction of this model is effectively evaluated. Through the analysis of the above experiments, the following conclusions are drawn:

1. The humanistic literacy evaluation of female higher vocational students is as high as 95%, and after the humanistic literacy course training and quality education, the evaluation scores of female students have improved significantly, and some scores can reach 100 points, and the level of quality of humanistic literacy is not directly linked to professional categories
2. Students over the age of 18 years old have good results, high evaluation scores, high support, and high reliability, and the data of male and female students reaches 80%. It can be concluded that the continuous growth of the school's young students is in line with the direction of the school's talent development

Pursuant to the above discussion, vocational colleges can guide higher vocational students to cultivate literacy in the aspects of team spirit, cooperation ability, spirit of overcoming difficulties, and perseverance, so that they can be further valued by employers and society. Therefore, in the future training path, it is necessary to firmly grasp the training standards of humanistic quality and strive to cultivate more comprehensive, modern, and high-quality vocational professionals.

## Figures and Tables

**Figure 1:** Data mining process.

**Figure 2:** Comparison of male and female students before and after optimization.

**Figure 3:** Comparison of 16-20-year-old students before and after optimization.

**Table 1:** Basic information of students.

Student ID	Student name	Age	Gender	Grade	Professional category
1	Student A	17	Female	Class of 2021	Food quality and safety
2	Student B	17	Male	Class of 2021	Electrical automation
3	Student C	18	Female	Class of 2020	Industrial design
4	Student D	19	Female	Class of 2020	Food quality and safety
5	Student E	18	Male	Class of 2020	Electrical automation
6	Student F	17	Female	Class of 2021	Food quality and safety
7	Student G	19	Male	Class of 2019	Electrical automation
8	Student H	18	Male	Class of 2021	Industrial design

## Data Availability

The dataset can be accessed upon request.
